# MiR-25-3p targets PTEN to regulate the migration, invasion, and apoptosis of esophageal cancer cells via the PI3K/AKT pathway

**DOI:** 10.1042/BSR20201901

**Published:** 2020-10-14

**Authors:** Liang Zhang, Zhuang Tong, Zhe Sun, Guolian Zhu, Erdong Shen, Yanfeng Huang

**Affiliations:** 1 Department of Thoracic Surgery, Cancer Hospital of China Medical University, Liaoning Cancer Hospital and Institute, Shenyang, Liaoning Province 110042, China; 2 Department of Surgical Oncology, First Affiliated Hospital of China Medical University, Shenyang, Liaoning Province 110001, China; 3 Department of Oncology, Shenyang Fifth People Hospital, Shenyang, Liaoning Province 110001, China; 4 Department of Oncology, Yueyang First People’s Hospital, Yueyang, Hunan 414000, China

**Keywords:** apoptosis, esophageal cancer, invasion, migration, miR-25-3p, PTEN

## Abstract

**Background:** Esophageal cancer (EC) is one of the most common malignant tumors of the digestive system. MiR-25-3p was proved to be a biomarker for the diagnosis and treatment of many cancers. MiR-25-3p was found to be high expressed in the blood of EC patients. The aim of the present study was to explore the effect of miR-25-3p and its target gene on EC.

**Methods:** miR-25-3p expression in the blood of EC patients and EC cells was detected by RT-qPCR. The target of miR-25-3p was identified by bioinformatics and luciferase reporter assay. After transfection, cell viability, apoptosis, migration, and invasion were detected by MTT, flow cytometry, wound healing, and transwell assays, respectively. The expressions of PTEN, Bax, Bcl-2, cleaved Caspase-3, p-PI3K, PI3K, p-AKT, and AKT were detected by Western blot.

**Results:** MiR-25-3p was high expressed in the blood of EC patients and EC cells. MiR-25-3p targeted PTEN and inhibited the expression of PTEN. MiR-25-3p mimic increased the viability, migration, invasion and the expressions of Bcl-2, and inhibited the apoptosis and the expression of Bax and cleaved caspase-3 in EC cells. MiR-25-3p mimic also enhanced the expressions of p-PI3K and p-AKT and the ratios of p-PI3K/PI3K and p-AKT/AKT in EC cells. PTEN overexpression not only had an opposite effect of miR-25-3p mimic, but also reversed the effect of miR-25-3p mimic on EC cells.

**Conclusion:** MiR-25-3p targeted PTEN to promote the migration and invasion, and inhibit apoptosis of EC cells via the PI3K/AKT pathway, which might provide a new therapeutic target for EC treatment.

## Introduction

Esophageal cancer (EC) is one of the most common malignant tumors of the digestive system and the sixth leading cause of cancer-related deaths in the world [1,2]. Globally, there are around more than 455,800 new cases and over 400,200 deaths of EC per year [1,3]. Owing that the symptoms of early EC patients are not obvious, a majority of EC patients are usually diagnosed at advanced stages [4,5]. Despite the innovative development of EC treatment in recent years, the 5-year survival rate of EC patients is still as low as 21% [1,6]. Like other cancers, the occurrence and progression of EC are closely related to the abnormal expressions of multiple genes, such as oncogenes, tumor-suppressor, and growth-related genes [5–8]. Therefore, the identification of cancer-related genes is greatly beneficial to developing novel therapeutic targets for the prevention and treatment of EC.

MicroRNAs (miRNAs) are endogenous, small (19–25 nucleotides) non-coding single-stranded RNA molecules, which play important roles in many biological processes [8–10]. More and more evidence has shown that abnormal expressions of miRNAs are highly related to the occurrence and progression of various diseases and cancers, including EC [10,11]. Recently, the abnormal expression level of miR-25-3p has been discovered in different diseases gradually. For instance, miR-25-3p was found to be up-regulated in triple-negative breast cancer, osteosarcoma, and gastric cancer [12–14]; while it was found to be down-regulated in acute-on-chronic liver failure and tongue squamous cell carcinoma [15,16]. In addition, miR-25-3p was proved to be a biomarker for the diagnosis and treatment of many cancers and able to regulate the biological functions of various cells [13,15]. Besides, miR-25-3p could enhance the proliferation and migration of glioma cells, impair tumorigenesis of gastric cancer and regulate the migration of gastric cancer cells, and promote the pre-metastatic niche formation of colorectal cancer [14,17,18]. miR-25-3p regulates cancer cell processes by targeting genes or regulatory signaling pathways [17,19,20]. Serum exosomal miR-25-3p may be as biomarkers for the detection of esophageal adenocarcinoma [21]. In addition, Zhang et al. predicted that miR-25-3p was high expressed in EC [5]. However, the expression level of miR-25-3p in EC has not been verified by other scholars as far as we know and whether miR-25-3p exerts a regulatory effect on EC cells need to be investigated.

Therefore, the purpose of the present study was to explore the role of miR-25-3p in EC and further investigate the potential mechanism. In our study, we found that miR-25-3p was high expressed in the blood of EC patients and EC cells. Moreover, miR-25-3p promoted the viability, migration and invasion, and inhibited the apoptosis via targeting PTEN by regulating PI3K/AKT signaling pathway in EC cells. This result might provide new promising therapeutic strategies for EC.

## Methods

### Serum samples

The blood of 40 EC patients and 40 healthy volunteers were gathered at Cancer Hospital of China Medical University, Liaoning Cancer Hospital and Institute between May 2018 and July 2019. The serum was collected from blood through centrifugation at 12000 rpm for 10 min, and then the serum was aliquoted and stored at −80°C until use. None of the patients had received chemotherapy or radiotherapy.

### Cell culture

Normal human esophageal epithelial cell line HET-1A (ml056593) was obtained from Mibio (https://www.mlbio.cn/search.php?keywords=HET-1A) (Shanghai, Chian); human EC cell lines including Eca-109, EC9706, OE19, and OE33 were obtained from Jennio (Guangzhou, China) (http://www.jennio-bio.com/); human EC cell line KYSE-150 (XY449) was obtained from X-Y Biotechnology (http://shxysw.bioon.com.cn/products.asp) (Shanghai, China); human EC cell line SKGT4 was obtained from Cobioer Biosciences (http://www.co-bioer.com/Products-23324910.html) (Nanjing, China). All cells were cultured in RPMI 1640 medium (72400120, Gibco, MA, U.S.A.) containing 10% fetal bovine serum (FBS; 16140071, Gibco) and incubated in a 37°C, humid atmosphere with 5% CO_2_.

### Transfection

MiR-25-3p mimic (miR10000081-1-5) and mimic control (MC; miR1N0000002-1-5) were obtained from RIBOBIO (Guangzhou, China). Plasmid-overexpressing PTEN, which was ligated into pcDNA3.1, was synthesized from GenePharma (Shanghai, China). The primer used to get the overexpression sequence of PTEN was shown as follows: F: 5′-TTTGAAGACCATAACCCACCAC-3′, R: 5′-ATTACACCAGTTCGTCCCTTTC-3′. Plasmids without any target sequence were used as negative control (NC).

Then, the plasmids were diluted with RNase-free H_2_O (ST876, Beyotime, Shanghai, China) and stored at −20°C for later use. Before transfection, Eca-109 and OE19 cells were plated into six-well plates, each well containing 1.0 × 10^6^ cells and 2 ml of complete medium. After the cells grew overnight until they reached 80% confluence, 100 μl of medium was added to dilute 2 μg of the plasmids, while 3 μl of lipofectamine 2000 (11668-019, Invitrogen, MA, U.S.A.) was added to another 100 μl of medium. After that, the two media were mixed and incubated for 15 min at room temperature. Finally, the mixed liquid was added into the cells of each well, and 1.8 ml of medium was then added into the cells and cultured for an additional 48 h.

### Luciferase reporter assay

The fragments of PTEN wild-type (PTEN-WT) (5′-AGTTCTAGAAATTTTGTGCAATA-3′) and PTEN mutant (PTEN-MUT) (5′-AGTTCTAGAAATTTTTACACGCA-3′) binding sites for miR-25-3p were inserted into pmirGLO luciferase Vectors (E1330, Promega, CA, U.S.A.). Eca-109 and OE19 cells were placed into 48-well plates, each well containing 3.0 × 10^4^ cells and 300 μl of complete medium. After growing overnight, these target vectors or non-target vectors were co-transfected with miR-25-3p mimic or mimic control into the cells using Lipofectamine 2000 for 48 h. Next, the cells were gathered to perform Dual-Luciferase Reporter Assay (Promega). Luciferase activity of the cells was determined using a GloMax fluorescence reader (Promega).

### MTT assay

MTT (B7777, APExBIO, Houston, U.S.A.) was used to test cell viability. After transfection, Eca-109 and OE19 cells were laid into 96-well plates, each well containing 1.0 × 10^4^ cells and 100 μl of complete medium. After growth for another 24, 48, or 72 h, the cells were incubated with MTT reagent (0.5 mg/ml) for 4 h. Then, the MTT solution was discarded and 100 μl of DMSO (ST038, Beyotime) was added to each well. Finally, the absorbance of each well was measured at 570 nm using a microplate reader (Infinite M200 PRO, Tecan Austria GmbH, Austria).

### Wound healing assay

After transfection, Eca-109 and OE19 cells were placed into six-well plates, each well containing 3.5 × 10^5^ cells and 2 ml of complete medium. The cells were cultured until they reached 95% confluence. Then, a vertical wound in each well was created using a 20 μl pipette tip, and a medium without FBS was added into each well. Images of each well were collected at 0 and 48 h with a phase-contrast optical microscope (Axio Lab.A1 pol; Leica, Solms, Germany). ImageJ software 1.8.0 (National Institutes of Health, Bethesda, U.S.A.) was used to analyze the images in this assay.

### Transwell assay

Transwell cell culture chambers were pre-coated with Matrigel (354234, Corning Life Sciences, NY, U.S.A.) and the chambers were placed into a 24-well plate. After transfection, Eca-109 and OE19 cells were pipetted into the chambers at a density of 2 × 10^5^ cells/well, which contained a suspension solution supplemented with 0.2 ml of medium without FBS, and then 0.7 ml of corresponding complete medium was added into the lower chamber. Afterwards, the cells were incubated for 48 h and the upper-side of the polycarbonate membrane was wiped off, leaving the underside of the membrane containing invaded cells. Finally, the cells were stained with Crystal Violet (C0121, Beyotime) for 15 min at room temperature. Three random areas on each membrane were chosen to count (×250) the cell number under a phase-contrast optical microscope (Axio Lab.A1 pol; Leica, Solms, Germany). ImageJ software 1.8.0 was used to analyze the images.

### Flow cytometry

The apoptosis of Eca-109 and OE19 cells was estimated using an Annexin V/PI kit (KGA108, KeyGen Biotech, Nanjing, China) through flow cytometry. In brief, after transfection, Eca-109 and OE19 cells were placed into six-well plates, each well containing 2.0 × 10^5^ cells and 2 ml of complete medium. After incubation for another 24 h, the cells were collected and incubated with Annexin V for 15 min at normal atmospheric temperature in the dark. Then, the cells were incubated with PI for 25 min at normal atmospheric temperature in the dark. Finally, the fluorescence intensity of the cells was measured using a fluorescence-activated cell sorting caliber (Cytoflex, Beckman Coulter, CA, U.S.A.), and the cell apoptosis was analyzed using CytExpert 2.0 software (Beckman Coulter).

### RNA extraction and RT-qPCR

MiRNAs were extracted from clinical samples and cultured cell lines using a MiRcute miRNA Isolation Kit (FP401, TIANGEN, Beijing, China). In brief, the samples and cells were collected into a 1.5 ml centrifugal tube (615001, Nest, Wuxi, China) and mixed with lysis buffer. Then, 200 μl of chloroform (C805334, Macklin, Shanghai, China) was added into the cells and the tube was shaken violently for 1 min. After resting for 5 min at room temperature, the cells were centrifuged for 20 min (13400 × ***g***) and then the miRNA solution was collected to a new 1.5 ml tube. The new tube was then added with ethanol and centrifuged for 15 min (13400 × ***g***). After centrifugation, the sediment was miRNA, and it was diluted with RNase-free H_2_O. Then, a PrimeScript RT Kit (RR037A, Takara, Dalian, China) was used to reverse-transcribe RNA into cDNA according to the instructions. Finally, gene expression was detected by RT-qPCR assay using a Verso 1-step RT-qPCR Kit (A15300, Thermo Scientific, MA, U.S.A.) in ABI 7500 Fast Real-Time PCR System (Applied Biosystems, CA, U.S.A.), and the condition of qPCR was set as: at 95°C for 30 s, at 60°C for 30 s, and 45 cycles of at 60°C for 30 s. RNA was quantified by the 2^−ΔΔCT^ method. The primer sequences were as follows: miR-25-3p-F: 5′-CATTGCACTTGTCTCGGTCTGA-3′, miR-25-3p-R: 5′-GCTGTCAACGATACGCTACGTAACG-3′; U6-F: 5′-CTCGCTTCGGCAGCACA-3′, U6-R: 5′-AACGCTTCACGAATTTGCGT-3′. Total RNA were extracted using TRIzol reagent (Invitrogen; Thermo Fisher Scientific, Inc.), and cDNA was synthesized using oligodT and SuperScript II reverse transcriptase (Invitrogen). The amplification of the RT-qPCR reaction was conducted using a SYBR Premix Ex Taq kit (Takara Bio, Inc.) in the 7500 real-time PCR system (Applied Biosystems), and the condition of qPCR was set as: at 95°C for 3 min, followed by 40 cycles at 95°C for 30 s and at 60°C for 30 s. The primer sequences were as follows: Bcl-2-F: 5′-TTGTGGCCTTCTTTGAGTTCGGTG-3′, Bcl-2-R: 5′-GGTGCCGGTTCAGGTACTCAGTCA-3′; Bax-F: 5′-CCTGTGCACCAAGGTGCCGGAACT-3′; Bax-R; 5′-CCACCCTGGTCTTGGATCCAGCCC-3′ PTEN-F: 5′-CCGAAAGGTTTTGCTACCATTCT-3′, PTEN-R: 5′-AAAATTATTTCCTTTCTGAGCATTCC-3′; GAPDH-F: 5′-GTCAACGGATTTGGTCTGTATT-3′, GAPDH-R: 5′-AGTCTTCTGGGTGGCAGTGAT-3′.

### Western blot assay

Total protein was isolated from the Eca-109 and OE19 cells using RIPA lysis buffer (P0013B, Beyotime), and a BCA Assay Kit (23250, Pierce, MA, U.S.A.) was used to determine the total protein concentration. Then, total protein (30 µg) was separated in each lane by 10% SDS-PAGE (P0052A, Beyotime), electro-blotted and transferred to NC membranes (HTS112M, Millipore, Billerica, MA, U.S.A.). Next, the membranes were incubated with 5% skimmed milk for 2 h at normal atmospheric temperature, and then incubated with the following primary antibodies: Bax (1:1000, 20kD, #5023, CST, CA, U.S.A.), Bcl-2 (1:1000, 26kD, #4223, CST), cleaved Caspase-3 (1:1000, 17kD, #9661, CST), PTEN (1:1000, 54kD, #9188, CST), p-PI3K (1:1000, 85kD, #4228, CST), PI3K (1:1000, 85kD, #4292, CST), p-AKT (1:1000, 60kD, #9271, CST), AKT (1:1000, 60kD, #4691, CST), and GAPDH (1:1000, 37kD, #5174, CST). The next day, HRP-conjugated secondary antibody goat anti-rabbit IgG (1:5000, ab205718, Abcam, CA, U.S.A.) or goat anti-mouse IgG (1:5000, ab205719, Abcam) was incubated with the membranes for 1 h at room temperature. Finally, SuperSignal West Pico Chemiluminescent Substrate (34078, Thermo Scientific, MA, U.S.A.) was used to incubate the membranes for detecting the signal. Image Lab™ Software (version 3.0) was used for densitometric analysis and quantification of the Western blot data (Bio-Rad Laboratories Inc., Hercules, CA, U.S.A.).

### Statistical analysis

Student’s *t*-test and one-way ANOVA were applied to analyze the data in the present study using SPSS software (version 18.0). LSD and Dunnet’s were used as post-hoc tests. The statistical data were expressed as mean ± standard deviation. All experiments were conducted three times. *P*<0.05 was considered as statistically significant.

## Results

### MiR-25-3p was high expressed in the blood of EC patients and EC cell lines and it increased the viability of Eca-109 and OE19 cells

We first analyzed the expression level of miR-25-3p in the blood of EC patients, and as shown in Figure 1A, miR-25-3p was high expressed in the blood of EC patients as compared with normal blood (*P*<0.001). We then detected the expression level of miR-25-3p in a serious of EC cell lines (Eca-109, EC9706, KYSE-150, SKTG4, OE19, and OE33) and the normal human esophageal epithelial cell line HET-1A (Figure 1B), and the results demonstrated that miR-25-3p was also high expressed in EC cells as compared with HET-1A cells (*P*<0.001). Considering that the expression of miR-25-3p in Eca-109 and OE19 cells was higher than in other cells, these two cell lines were chosen for later use. After we transfected miR-25-3p mimic into Eca-109 and OE19 cells, the transcription level of miR-25-3p was obviously increased as compared with the MC groups (*P*<0.001; Figure 1C,D). Then we detected the effects of miR-25-3p on the viability of these two cells (Figure 1E,F), and the results indicated that miR-25-3p mimic significantly increased the viability of Eca-109 and OE19 cells after culture for 48 and 72 h as compared with the MC group (*P*<0.05).

**Figure 1:** MiR-25-3p was high expressed in the blood of EC patients and EC cell lines and it increased the viability of Eca-109 and OE19 cells (**A**) The expression level of miR-25-3p in the blood of EC patients was detected by RT-qPCR. U6 was used as an internal control (^###^*P*<0.001, vs. normal). (**B**) The expression level of miR-25-3p in EC cell lines (Eca-109, EC9706, KYSE-150, SKTG4, OE19, and OE33) and normal human esophageal epithelial cell line (HET-1A) was analyzed by RT-qPCR. U6 was used as an internal control (***P<0.001, vs. HET-1A). (**C** and** D**) The transfection efficiency of miR-25-3p mimic in Eca-109 and OE19 cells was detected by RT-qPCR. U6 was used as an internal control (^∧∧∧^*P*<0.001, vs. MC). (**E** and **F**) The viability of Eca-109 and OE19 cells after transfection of miR-216a-3p mimic was detected by MTT assay (^∧^*P*<0.05, ^∧∧^*P*<0.01, vs. MC). All experiments were conducted three times. (EC: esophageal cancer, M: miR-25-3p mimic, MC: mimic control).

### MiR-25-3p mimic inhibited the apoptosis and promoted the migration and invasion of Eca-109 and OE19 cells and regulated the expressions of apoptosis-related factors in Eca-109 and OE19 cells

Then we detected the effects of miR-25-3p on the apoptosis of Eca-109 and OE19 cells, and the results indicated that miR-25-3p mimic significantly decreased the relative apoptosis rates of Eca-109 and OE19 cells as compared with the MC group (*P*<0.001; Figure 2A–D). Mechanically, we further detected the expressions of apoptosis-related factors in Eca-109 and OE19 cells. The results exhibited that miR-25-3p mimic inhibited the protein expressions of Bax and Cleaved caspase-3 and up-regulated the expression of Bcl-2 in Eca-109 and OE19 cells as compared with the MC group (*P*<0.001; Figure 2E,F,I,J). The result also showed that miR-25-3p mimic promoted the mRNA expression of Bcl-2, but inhibited Bax mRNA expression (*P*<0.001; Figure 2G,H). In addition, we detected the changes of migration and invasion of Eca-109 and OE19 cells after transfection of miR-25-3p mimic. As shown in Figure 3, the relative migration and invasion rates of Eca-109 and OE19 cells were both significantly increased by miR-25-3p mimic (*P*<0.001), which indicated that miR-25-3p could enhance the migration and invasion abilities of Eca-109 and OE19 cells.

**Figure 2:** MiR-25-3p mimic inhibited the cell apoptosis through regulating the expressions of apoptosis-related factors in Eca-109 and OE19 cells (**A–D**) The apoptosis of Eca-109 and OE19 cells after transfection of miR-25-3p mimic was detected by flow cytometry. (**E** and **F**) The protein expressions of Bcl-2, Bax, and Cleaved caspase-3 in Eca-109 after transfection of miR-25-3p mimic were detected by Western blot. (**G** and **H**) The mRNA expressions of Bcl-2 and Bax in Eca-109 and OE19 cells were detected by RT-qPCR. (**I** and** J**) The protein expressions of Bcl-2, Bax, and Cleaved caspase-3 in OE19 cells after transfection of miR-25-3p mimic were detected by Western blot. All experiments were conducted three times (^∧∧^*P*<0.01, ^∧∧∧^*P*<0.001, vs. MC). (M: miR-25-3p mimic, MC: mimic control).

**Figure 3:** MiR-25-3p mimic promoted the migration and invasion of Eca-109 and OE19 cells (**A** and** B**) The migration of Eca-109 and OE19 cells after transfection of miR-25-3p mimic was detected by wound healing assay. (**C** and **D**) The invasion of Eca-109 and OE19 cells after transfection of miR-25-3p mimic was detected by transwell assay. All experiments were conducted three times (^∧∧^*P* < 0.01, ^∧∧∧^*P* < 0.001, vs. MC). (M: miR-25-3p mimic, MC: mimic control).

### PTEN was targeted by miR-25-3p and it reversed the inhibitory effect of miR-25-3p mimic on the expression of PTEN in Eca-109 and OE19 cells

The analysis results of Targetscan7.2 predicted that PTEN was a target of miR-25-3p owing that miR-25-3p contained sequences complementary to PTEN-WT (Figure 4A). In order to verify this prediction, we conducted luciferase reporter assay, and as shown in Figure 4B,C, luciferase activity was decreased in both Eca-109 and OE19 cells that were co-transfected with miR-25-3p mimic and PTEN-WT as compared with that in the blank groups (*P*<0.001); while there was no difference in the luciferase activity between the blank groups and the Eca-109 and OE19 cells co-transfected with miR-25-3p mimic and PTEN-MUT, which verified that PTEN could be targeted by miR-25-3p. Furthermore, as shown in Figure 4D–G, the protein expression of PTEN in these two cells was up-regulated by PTEN overexpression and down-regulated by miR-25-3p mimic as compared with the NC group (*P*<0.01); while after co-overexpression of miR-25-3p and PTEN (M+PTEN group), the inhibitory effect of miR-25-3p on PTEN expression was reversed by PTEN overexpression as compared with the M and M+NC groups, though the expression of PTEN was still lower than that in the PTEN group. In addition, the mRNA expression of PTEN in these two cells was up-regulated by PTEN overexpression and down-regulated by miR-25-3p mimic as compared with the NC group, and the inhibitory effect of miR-25-3p on PTEN expression was reversed by PTEN overexpression (*P*<0.01; Figure 4H,I).

**Figure 4:** PTEN was targeted by miR-25-3p and it reversed the regulatory effect of miR-25-3p mimic on the expression of PTEN and the viability of Eca-109 and OE19 cells (**A**) The putative binding site between PTEN and miR-25-3p was predicted by Targetscan7.2. (**B** and **C**) The results of luciferase assay validated that PTEN was targeted by miR-25-3p in Eca-109 and OE19 cells (^†††^*P*<0.001, vs. Blank). (**D**–**G**) The protein expression level of PTEN in Eca-109 and OE19 cells was analyzed by Western blot. GAPDH was used as an internal control. (**H and I**) The mRNA expression level of PTEN in Eca-109 and OE19 cells was analyzed by RT-qPCR. (**J and K**) The viability of Eca-109 and OE19 cells was analyzed by MTT assay. All experiments were conducted three times (^∧∧^*P* < 0.01, ^∧∧∧^*P* < 0.001, vs. NC; ^###^*P* < 0.001, vs. PTEN; ***P < 0.001, vs. M; ^ΔΔΔ^*P* < 0.001, vs. M+NC) (WT: wild type, MUT: mutation, M: miR-25-3p mimic, MC: mimic control, NC: negative control).

### PTEN reversed the promoting effect of miR-25-3p mimic on the viability, migration, and invasion of Eca-109 and OE19 cells

As shown in Figure 4J,K, the viability of Eca-109 and OE19 cells was enhanced by miR-25-3p mimic and inhibited by PTEN overexpression as compared with the NC group (*P*<0.001); while after co-overexpression of miR-25-3p and PTEN (M+PTEN group), the promoting effect of miR-25-3p mimic on cell viability was reversed by PTEN overexpression as compared with the M and M+NC groups, though the cell viability was still higher than that in the PTEN group (*P*<0.001). We further detected the migration and invasion of Eca-109 and OE19 cells. As shown in Figure 5, the relative migration and invasion rates of Eca-109 and OE19 cells were enhanced by miR-25-3p mimic and inhibited by PTEN overexpression as compared with the NC group (*P*<0.001); while after co-overexpression of miR-25-3p and PTEN (M+PTEN group), the promoting effect of miR-25-3p mimic on cell migration and invasion was reversed by PTEN overexpression as compared with the M and M+NC groups, though the relative cell migration and invasion rates were still higher than those in PTEN group (*P*<0.001).

**Figure 5:** PTEN reversed the promoting effect of miR-25-3p mimic on the migration and invasion of Eca-109 and OE19 cells (**A**–**D**) The migration of Eca-109 and OE19 cells after transfection was detected by wound healing assay. (**E**–**H**) The invasion of A549 and H1975 cells after transfection was detected by transwell assay. All experiments were conducted three times (^∧∧∧^*P*<0.001, vs. NC; ^###^*P*<0.001, vs. PTEN; ***P<0.001, vs. M; ^ΔΔΔ^*P*<0.001, vs. M+NC). (WT: wiid type, MUT: mutation, M: miR-25-3p mimic, MC: mimic control, NC: negative control)

### PTEN reversed the effect of miR-25-3p mimic on inhibiting cell apoptosis and promoting the activation of the PI3K/AKT pathway in Eca-109 and OE19 cells

As shown in Figure 6A,B, the apoptosis of Eca-109 and OE19 cells was suppressed by miR-25-3p mimic and enhanced by PTEN overexpression as compared with the NC group (*P*<0.05); while after co-overexpression of miR-25-3p and PTEN (M+PTEN group), the inhibitory effect of miR-25-3p mimic on cell apoptosis was reversed by PTEN overexpression as compared with the M, M+NC, and PTEN groups (*P*<0.001). What’s more, as shown in Figure 6C–F, the expressions of p-PI3K and p-AKT in Eca-109 and OE19 cells were enhanced by miR-25-3p mimic and inhibited by PTEN overexpression as compared with the NC group (*P*<0.001); while after co-overexpression of miR-25-3p and PTEN (M+PTEN group), the promoting effect of miR-25-3p mimic on the expressions of p-PI3K and p-AKT was reversed by PTEN overexpression as compared with the M, M+NC, and PTEN groups (*P*<0.001). Although the expressions of PI3K and AKT in Eca-109 and OE19 cells were not changed, the ratios of p-PI3K/PI3K and p-AKT/AKT exhibited the same tendency as p-PI3K and p-AKT did among these groups in both Eca-109 and OE19 cells (*P*<0.001; Figure 6G–J), which further revealed that PTEN reversed the promoting effect of miR-25-3p mimic on the activation of the PI3K/AKT pathway.

**Figure 6:** PTEN reversed the effect of miR-25-3p mimic on inhibiting cell apoptosis and promoting the activation of the PI3K/AKT pathway in Eca-109 and OE19 cells (**A** and** B**) The apoptosis of Eca-109 and OE19 cells after transfection was detected by flow cytometry. (**C**–**F**) The expression of p-PI3K, PI3K, p-AKT, and AKT in Eca-109 and OE19 cells after transfection were detected by Western blot, GAPDH was used as an internal control. (**G–J**) The ratio of p-PI3K/PI3K and p-AKT/AKT of the Western blot results in Eca-109 and OE19 cells was calculated. All experiments were conducted three times (^∧∧∧^*P* < 0.001, vs. NC; ^###^*P* < 0.001, vs. PTEN; **P < 0.01, ***P < 0.001, vs. M; ^ΔΔ^*P* < 0.01, ^ΔΔΔ^*P* < 0.001, vs. M+NC). (WT: wild type, MUT: mutation, M: miR-25-3p mimic, MC: mimic control, NC: negative control)

## Discussion

In the present study, we first found that miR-25-3p was high expressed in the blood of EC patients and EC cells. Then we revealed that miR-25-3p targeted PTEN and that miR-25-3p mimic increased the viability, migration and invasion and inhibited the apoptosis of EC cells while enhancing the activation of the PI3K/AKT pathway. PTEN had an opposite effect of miR-25-3p mimic and further reversed the effect of miR-25-3p mimic on EC cells, which further verified that miR-25-3p could target PTEN to regulate the migration, invasion, and apoptosis of EC cells via the PI3K/AKT pathway. Our study identified that miR-25-3p might serve as a novel candidate biomarker for the detection and therapy of EC.

Recently, more and more evidence has confirmed that abnormal expressions of miRNAs are closely associated with the occurrence and progression of different kinds of cancers and most of these abnormally expressed miRNAs could be used as biomarkers for the diagnosis and therapy of many cancers [7,9,22]. For instance, miR-215-5p was lowly expressed in prostate cancer tissues and cells [23]; miR-182-5p was highly expressed in non-small cell lung cancer [24]; miR-96 was up-regulated in ovarian cancer [25]. As for EC, research has found that miR-486 was down-regulated in EC tissues and cells while miR-873 was up-regulated. In addition, miR-486 and miR-873 were proved to have a regulatory effect on EC cells and could be further used as biomarkers for EC diagnosis [1,4]. Recently, it has been predicted that miR-25-3p was highly expressed in EC tissues [5]. In the present study, we not only found that miR-25-3p was up-regulated in the blood of EC patients and cells but also revealed that miR-25-3p had the ability to promote the migration and invasion and inhibited the apoptosis of EC cells, which indicated that miR-25-3p played a crucial role in the progression of EC, though the potential mechanism still needs further investigation.

An increasing number of studies have proved that miRNAs could target certain mRNAs and further regulate the progression of a serious diseases [26,27]. Some targets have been proved to be targeted by miR-25-3p in different kinds of diseases. For instance, BTG2 was targeted by miR-25-3p to promote the proliferation of breast cancer [12]; FBXW7 and DKK3 could be targeted by miR-25-3p to enhance the proliferation and migration of glioma cancer cells [17]. In the present study, we further found that PTEN was targeted by miR-25-3p in EC cells. PTEN, which was identified in 1977, is a classical cancer suppressor and possesses lipid and protein phosphatase activities [28]. In malignant cells, PTEN has been shown to be silenced by the expressions of a number of micro-RNAs and able to drive a transcriptional program that is essential for maintaining the malignant state of diseases, such as cell proliferation, apoptosis, invasion, and adhesion [29,30]. Shi et al. reported that PTEN was targeted by miR-17-5p to regulate the proliferation and autophagy of thyroid cancer [30]; Chen et al. proved that miR-21 regulated the proliferation and apoptosis of bladder cancer mediated through PTEN [31]; PTEN was also targeted by miR-216a to enhance the proliferation and fibrogenesis of human cardiac fibroblasts [32]. Similarly, in the present study, we found that PTEN not only inhibited the migration and invasion, and induced apoptosis of EC cells, but also reversed the effect of miR-25-3p on EC cells, which further confirmed that miR-25-3p regulated the migration, invasion, and apoptosis of EC cells by targeting PTEN. It's also well known that the activity of PTEN antagonizes the PI3K/AKT pathway to suppress cancer cell survival, which means that deficient PTEN expression leads to the PI3K/AKT pathway activation, thereby enhancing cell anti-apoptosis [33–35]. In investigating the down-stream mechanism of miR-25-3p mediated in EC in the present study, we also observed that enhanced PTEN expression suppressed the activation of the PI3K/AKT pathway, and miR-25-3p-induced decrease of PTEN expression further enhanced the PI3K/AKT pathway activation, while overexpression of PTEN could inhibit the effect of miR-25-3p on this pathway.

## Conclusion

In conclusion, this research revealed that miR-25-3p enhanced the migration, invasion and suppressed the apoptosis of EC cells through PTEN-mediated PI3K/AKT pathway, which indicated that miR-25-3p might be a target for EC treatment.

## Abbreviations

AKT: protein kinase B
Bax: Bcl-2-associated X
Bcl-2: B-cell lymphoma-2
EC: esophageal cancer
miRNA: microRNA
PI3K: phosphatidylinositol 3 kinase
PTEN: phosphatase and tensin homologue deleted on chromosome10
